The article "Cationic solid lipid nanoparticles loaded by integrin β1 plasmid DNA attenuates IL-1β-induced apoptosis of chondrocyte" was retracted in 2023. Reasons: plagiarized images; duplicated images; overlap with other authors' work; signs of a paper mill.

# Cationic solid lipid nanoparticles loaded by integrin β1 plasmid DNA attenuates IL-1β-induced apoptosis of chondrocyte

**DOI:** 10.18632/aging.103656

**Published:** 2020-11-27

**Authors:** Yuejiang Zhao, Hanwen Chen, Lu Wang, Zhiyuan Guo, Shijie Liu, Simin Luo

**Affiliations:** 1 The First Department of Orthopedics, Cangzhou Central Hospital, Cangzhou, Hebei Province, China; 2 Department of Joint Surgery, Xingtan Hospital Affiliated to Shunde Hospital of Southern Medical University, Foshan, Guangdong Province, China; 3 Department of Bone and Joint Surgery, The First Affiliated Hospital, Jinan University, Guangzhou, Guangdong Province, China

**Keywords:** osteoarthritis, integrin β1, cationic solid lipid nanoparticles, chondrocytes

## Abstract

Aging-related inflammation is tightly linked with the development of osteoarthritis (OA). As the pro-inflammatory cytokine, IL-1β has been associated with physical dysfunction and frailty. It is still elusive whether and how IL-1β blockade improves the outcome of OA. Here we develop a cationic solid lipid nanoparticles (SLNs) system that effectively mediate non-viral delivery of plasmid DNA (pDNA) into cells. Compared with other DNA transfer technologies including lipofetamin 2000, SLNs-pDNA system is less toxic and exerts identical effectiveness on DNA transfer. Loaded with integrin β1 overexpression pDNA, the SLNs-pDNA mainly localized in cytoplasm and enforced expression of integrin β1 in rat chondrocytes. Moreover, upon exposure to IL-1β stimulation, SLNs-pDNA treatment attenuates the apoptosis rat chondrocytes and augments tissue repair. Our data thus demonstrate that SLNs-pDNA functions as a potential therapeutic nanomedicine in the treatment of osteoarthritis.

## INTRODUCTION

As a degenerative inflammatory disease, osteoarthritis (OA) is a common and frequently-occurring articular cartilage disease in the elderly, and usually responsible for joint pain and high rates of disability [1]. It is characterized by cartilage degenerative damage, such as the degradation of the cartilage matrix and the death of chondrocytes [2]. However, due to poor understanding for the pathogenesis of OA, there is currently a lack of effective interventions and treatments available to suppress disease progression such as restoring degraded cartilage [3, 4]. Although the drug treatments for OA have achieved the intensive progress, unsatisfactory prognosis still exist [5]. Thus, it is essential to search for effective strategies for the treatment of OA.

The unique cells in articular cartilage, chondrocytes, are involved in the synthesis and regulation of extracellular matrix (ECM), which play important role in the pathogenesis of OA [6, 7]. Accumulating evidence has shown that inhibiting apoptosis and promoting proliferation of chondrocytes may be crucial in the prevention and control of OA [8]. As a type of important surface adhesion receptors, integrin mainly mediate the adhesion between cells and ECM, and regulate various cell physiological processes, including growth, differentiation, proliferation, adhesion, and apoptosis [9–11]. Especially, integrin β1 can function as one major surface receptor in chondrocytes, which can interact with ECM, thereby regulating the differentiation, proliferation and apoptosis of chondrocytes by regulating cell signaling pathway [12–14]. However, few studies have evaluated whether integrin β1 can be a potential target for OA progression.

The article "Cationic solid lipid nanoparticles loaded by integrin β1 plasmid DNA attenuates IL-1β-induced apoptosis of chondrocyte" was retracted in 2023. Reasons: plagiarized images; duplicated images; overlap with other authors' work; signs of a paper mill.

Currently, solid lipid nanoparticles (SLNs) are reported to be a promising drug delivery system, and widely applied in disease therapy, due to its favorable properties such as high biocompatibility and transfection efficiency [15, 16]. Notably, previous studies have demonstrated that cationic SLNs can effectively mediate non-viral delivery of plasmid DNA (pDNA) into cells [17–19]. Therefore, in the current research, we developed the integrin β1 overexpression pDNA-loaded SLNs (SLNs-pDNA), and then characterization was detected. In addition, the effects of SLNs-pDNA on proliferation and apoptosis of IL-1β-induced chondrocytes were unraveled, which may be conducive to the prevention and control of OA.

## RESULTS

### Characterization of cationic solid lipid nanoparticles (SLNs)

Using transmission electronic microscope (TEM), all cationic SLNs were stable, uniform and spherical in shape, with ~200 nm of diameter (Figure 1A). Moreover, excellent homogeneity of cationic SLNs with the similar size of around 200 nm was measured by dynamic light scattering (DLS) assay (Figure 1B). As shown in Figure 1C, a negative average zeta potential of cationic SLNs was ~15 mV.

**Figure 1:** **Characterization of solid lipid nanoparticles (SLNs).** (**A**) The representative images of SLNs using transmission electron microscopy. (**B**) The size distribution of SLNs. (**C**) The zeta potential distribution of SLNs.

### Preparation of SLNs-pDNA system

To validate the capacity of SLNs that loaded plasmid DNA (pDNA), we used Gel retardation assay to assess the status of naked pDNA in presence or absence of SLNs. As shown in Figure 2A, in contrast to the typical supercoiled band of naked pDNA, the intensity of DNA band was attenuated along with the increased ratio of cationic SLNs to pDNA (Figure 2A). Furthermore, the electrophoretic mobility was ceased when the mass ratio was ≥ 4:1, which suggested that almost all the pDNA were integrated with cationic SLNs (Figure 2A). To study the efficacy of cationic SLNs on DNA transfer, we used the plasmid contains the gene encoding green fluorescent protein (GFP) and integrin β1 to couple with cationic SLNs or combine with Lipofectamine2000. As shown in Figure 2B, similar proportion of GFP^+^ cells were detected between the cationic SLNs-pDNA treated cells and the cells transfected with pDNA by Lipofectamine2000. To determine the subcellular localization of cationic SLNs-pDNA in rat chondrocytes, we performed the con-focal assay. As shown in Figure 2C, SLNs-pDNA were transferred into rat chondrocytes, and SLNs-pDNA did not co-locate with lysosomes. Using the qRT-PCR and western blot assays, both mRNA and protein levels of integrin β1 were obviously elevated in cells treated with SLNs-pDNA compared with cells treated with SLNs (control cells) (Figure 2D, *p* < 0.05). Our data thus validate the effectiveness of SLNs-pDNA system.

The article "Cationic solid lipid nanoparticles loaded by integrin β1 plasmid DNA attenuates IL-1β-induced apoptosis of chondrocyte" was retracted in 2023. Reasons: plagiarized images; duplicated images; overlap with other authors' work; signs of a paper mill.

**Figure 2:** **Identification of solid lipid nanoparticles-integrin β1 overexpression plasmid (SLNs-pDNA).** (**A**) Gel retardation assay of naked pDNA and SLNs/pDNA complexes with the different mass ratio. (**B**) Fluorescent microscopy of rat chondrocytes transfected by pDNA (Lipofectamine2000) and SLNs-pDNA. (**C**) Intracellular distribution assay of SLNs-pDNA in rat chondrocytes. (**D**) The mRNA and protein levels of integrin β1 in cells treated with SLNs-pDNA using qRT-PCR and western blot assays, respectively.

### *SLNs*-pDNA exhibits little cytotoxicity of rat chondroc*ytes*

*SLNs-pDNA* treatment exhibited little effects on cell viability (Figure 2B). To further confirm this result, we employed CCK-8 assay investigate the effects of *SLNs-pDNA* on cell proliferation. As shown in Figure 3, compared with normal control cells, Lipofectamine2000 exhibited remarkable toxic effects on rat chondrocytes. Although high dose of SLNs-pDNA also elicited mild cytotoxicity, low dose of SLNs-pDNA was non-toxic to rat chondrocytes (Figure 3).

**Figure 3:** **Solid lipid nanoparticles-integrin β1 overexpression plasmid (SLNs-pDNA) exhibited low cytotoxicity in rat chondrocytes.** Cell viability of rat chondrocytes transfected by pDNA (Lipofectamine2000) or different doses of SLNs-pDNA using CCK-8 assay.

### Effect of SLNs-pDNA on cell proliferation in IL-1β-induced rat chondrocytes

As the key pro-inflammatory cytokine, IL-1β was reported to induce apoptosis of rat chondrocytes and exacerbate the tissue damage. Consistent to the previous report, IL-1β treatment significantly limited cell viability (model group) compared with control cells (Figure 4A). To investigate whether SLNs-pDNA treatment affects this process, we pre-treated cells with SLNs-pDNA for 12hrs, then stimulated with IL-1β. As shown in Figure 4A, SLNs-pDNA treatment obviously increased cell resistance to IL-1β stimulation (*p* < 0.05). In addition, BrdU assay also revealed that IL-1β treatment (model group) remarkably inhibited the percentage of BrdU-positive cells, while SLNs-pDNA pretreatment elevated the percentage of BrdU-positive cells in IL-1β-induced rat chondrocytes (Figure 4B, *p* < 0.05). These results thus indicate that SLNs-pDNA sustains the survival of rat chondrocytes under IL-1β stimulation.

The article "Cationic solid lipid nanoparticles loaded by integrin β1 plasmid DNA attenuates IL-1β-induced apoptosis of chondrocyte" was retracted in 2023. Reasons: plagiarized images; duplicated images; overlap with other authors' work; signs of a paper mill.

**Figure 4:** **Solid lipid nanoparticles-integrin β1 overexpression plasmid (SLNs-pDNA) promoted cell proliferation in IL-1β-induced rat chondrocytes.** (**A**) Cell viability of rat chondrocytes treated with IL-1β (model group), or IL-1β + SLNs-pDNA (SLNs-pDNA group) using CCK-8 assay. (**B**) The percentage of BrdU-positive cells in rat chondrocytes treated with IL-1β (model group), or IL-1β + SLNs-pDNA (SLNs-pDNA group) using BrdU assay. *P < 0.05

### Effect of SLNs-pDNA on cell apoptosis in IL-1β-induced rat chondrocytes

To determine whether SLNs-pDNA blocks IL-1β-mediated cell death, we assessed the mitochondrial membrane potential by analyzing the status of JC-1. As shown in Figure 5A, majority of control cells presented JC-1 aggregates (red fluorescence) under quiescent condition, while increased JC-1 monomers (green fluorescence) and reduced JC-1 aggregates were observed in cells treated with IL-1β (model group) (Figure 5A). Notably, compared with cells treated with IL-1β, reduced level of JC-1 monomers and increased JC-1 aggregates were detected in cells pre-treated SLNs-pDNA (Figure 5A). In addition, flow cytometry analysis found that, compared with control cells, the stimulatory effects of IL-1β on apoptosis was attenuated by presence of SLNs-pDNA (Figure 5B, *p* < 0.05). We then performed western blot assay to detect the expression of apoptosis-related proteins, including cleaved caspase-3, and cleaved caspase-9. As shown in Figure 5C, compared with control cells, IL-1β treatment remarkably increased the expression of cleaved caspase-3, and cleaved caspase-9 (model group). Reciprocally, the presence of SLNs-pDNA exhibited opposite effects and downregulated the protein levels of cleaved caspase-3, and cleaved caspase-9 (Figure 5C, *p* < 0.05).

**Figure 5:** **Solid lipid nanoparticles-integrin β1 overexpression plasmid (SLNs-pDNA) inhibited cell apoptosis in IL-1β-induced rat chondrocytes**. (**A**) The mitochondrial membrane potential of rat chondrocytes treated with IL-1β (model group), or IL-1β + SLNs-pDNA (SLNs-pDNA group). (**B**) Cell apoptosis rate in rat chondrocytes treated with IL-1β (model group), or IL-1β + SLNs-pDNA (SLNs-pDNA group) by flow cytometry analysis. (**C**) The expression of apoptosis-related proteins, including cleaved caspase-3, and cleaved caspase-9 in rat chondrocytes treated with IL-1β (model group), or IL-1β + SLNs-pDNA (SLNs-pDNA group) by western blotting. *P < 0.05.

The article "Cationic solid lipid nanoparticles loaded by integrin β1 plasmid DNA attenuates IL-1β-induced apoptosis of chondrocyte" was retracted in 2023. Reasons: plagiarized images; duplicated images; overlap with other authors' work; signs of a paper mill.

## DISCUSSION

In the present study, we have developed a novel gene transfer system, SLNs-pDNA. Compared with Lipofectamine2000, SLNs-pDNA exhibited little cytotoxicity while similar transfection efficiency of pDNA in rat chondrocytes. In addition, IL-1β treatment significantly inhibited cell viability and the percentage of BrdU-positive cells, while increased cell apoptosis rate and disrupted mitochondrial membrane potential; however, SLNs-pDNA treatment reversely promoted cell proliferation and reduced cell apoptosis in IL-1β-induced rat chondrocytes.

Cationic SLNs have widely used for various biomedical applications due to their unique physiochemical properties, and the biocompatibility and safety of cationic SLNs are considered as key factors in biomedical applications. Several studies have evaluated the cytotoxicity of pDNA-loaded SLNs *in vitro* experiments. Penumarthi A et al. have reported that pDNA-loaded SLNs show low cytotoxicity and high transfection efficiency comparable to lipofectamine in dendritic cells [17]. Doroud D et al. also have revealed low cytotoxicity and transfection efficiency of cysteine proteinases gene-loaded ALNs in COS-7 cells [20]. In this study, we also found that SLNs-pDNA treatment exhibited low cytotoxicity and satisfactory transfection efficiency compared to the mediation of Lipofectamine2000. In addition, we also revealed the uptake of SLNs-pDNA in rat chondrocytes; however, SLNs-pDNA did not co-locate with lysosomes, indicating that SLNs might be able to protect the pDNA from degradation by lysosomes. All these results supported the no apparent cytotoxicity effect and biocompatibility of SLNs-pDNA *in vitro*.

It is well-known that chondrocytes play important roles in the occurrence and progression of OA, and increasing evidence has reported that targeting chondrocytes is suggested to be a critical strategy to alleviate OA [8, 21]. For examples, Wang et al. have documented that miR-142-3p is able to relieve the development of OA by inhibiting chondrocyte apoptosis and inflammation in OA via targeting the high mobility group box 1-mediated NF-kB signaling pathway [22]. Li et al. report that lncRNA plasmacytoma variant translocation 1 may be a potential therapeutic target for OA by regulating the apoptosis of chondrocytes [23]. In this study, we investigated the effect of SLNs-pDNA (integrin β1) on IL-1β-induced rat chondrocytes. Integrin β1 has been proved to exert important roles in regulating chondrocytes mechano-transduction and homeostasis [24]. It has been reported that integrin β1 is lowly expressed in OA chondrocytes [25], and the lack of integrin β1 in chondrocytes can cause cartilage hypoplasia and lead to multiple abnormalities of the joints [13]. Thus, this study upregulated the expression of integrin β1 by SLNs-pDNA treatment in rat chondrocytes, and we found that SLNs-pDNA treatment promoted cell viability and the percentage of BrdU-positive cells in IL-1β-induced rat chondrocytes, meanwhile, inhibited cell apoptosis rate and disrupted mitochondrial membrane potential. In addition, SLNs-pDNA treatment remarkably decreased the protein levels of cleaved caspase-3 and cleaved caspase-9 in IL-1β-induced rat chondrocytes. As a key downstream molecule of apoptosis pathway, caspase-3 can inhibit the ratio of Bcl-2/Bax and then contribute to cell apoptosis [26]. In addition, caspase-3 also can be activated followed by the recruitment and activation of caspase-9, thereby inducing cell apoptosis [27]. Therefore, we speculated that SLNs-pDNA might be able to decelerate the development of OA by promoting proliferation and inhibiting apoptosis of chondrocytes.

The article "Cationic solid lipid nanoparticles loaded by integrin β1 plasmid DNA attenuates IL-1β-induced apoptosis of chondrocyte" was retracted in 2023. Reasons: plagiarized images; duplicated images; overlap with other authors' work; signs of a paper mill.

In conclusion, this study successfully develop SLNs-pDNA system, and the treatment of SLNs-pDNA promotes cell proliferation and inhibits IL-1β-induced apoptosis of chondrocytes by overexpressing integrin β1. Overall, SLNs-pDNA might be a promising therapeutic nanomedicine in OA; however, the further *in vivo* experiments should be investigated.

## MATERIALS AND METHODS

### Preparation of cationic SLNs and SLNs-pDNA

The cationic SLNs were prepared using multiple emulsion method. In brief, 50 mg of stearic acid and 10 mg of lecithin were added into 1 mL of dichloromethane, and the solution was dissolved by ultrasound to form an oil phase. Then 50 μL of double distilled water was added into the oil phase, and W/O/W type colostrum was formed after sonicated for 2 min. Afterwards, colostrum was added into 10 mL solution containing 0.1% cetyl trimethyl ammonium bromide (CTAB), and stirred at high speed for 2.5 min until W/O/W type emulsion was formed. The obtained emulsion was dispersed into 40 mL solution containing 0.1% CTAB, and continue stirring for 12 h to completely evaporate the organic solvent. Lastly, the blank cationic SLNs suspension was obtained by filtering through polycarbonate membrane (0.45 μm of pore size), and the pH of the suspension was adjusted to 7.2-7.4. In addition, integrin β1 overexpression pDNA (GFP) (provided by GeneChem, Shanghai, China) were incubated with SLNs for 40 min at room temperature, thereby obtaining SLNs-pDNA.

The article "Cationic solid lipid nanoparticles loaded by integrin β1 plasmid DNA attenuates IL-1β-induced apoptosis of chondrocyte" was retracted in 2023. Reasons: plagiarized images; duplicated images; overlap with other authors' work; signs of a paper mill.

### Characterization of cationic SLNs

The morphological characteristics and particle size parameters of cationic SLNs were observed by transmission electron microscope (TEM) and dynamic light scattering (DLS). Briefly, the cationic SLNs solution was dripped onto a carbon-coated copper mesh for 2 min. After water evaporation, the sample was counterstained with 2% phosphotungstic acid for 2 min. Ultimately, the sample was observed by TEM (Tecnai G2 20 S-TWIN, FEI, Eindhoven, Netherlands). DLS of cationic SLNs was performed by Zetasizer Nano Z (Worcestershire, UK).

### Gel retardation assay

The formation and charge properties of SLNs-pDNA were by observed gel retardation assay, which might evaluate the effect of the amounts of nanoparticles on complex formation. Briefly, the complexes of SLN and pDNA (0.2 μg) with a mass ratio of 1:1, 2:1, 4:1, 6:1, and 8:1 as well as naked pDNA were subjected to electrophoretic analysis with 0.8% agarose gel (100 V, 30 min), and then observed by a UV transilluminator at 245 nm.

### Cell culture and treatment

Rat chondrocytes were provided by Procell (Wuhan, China), and maintained in DMEM (Gibco) with 10% fetal bovine serum (Gibco) under 37°C and 5% CO_2_. In order to mimic OA model, rat chondrocytes were cultured in serum-free medium containing 10 ng/mL IL-1β for 24 h. Subsequently, cells were treated with SLNs-pDNA for another 24 h.

### *In vitro* transfection assay

Rat chondrocytes were grown in 24-well plates for 24 h. After growing to 70% of confluence, cells were incubated with SLNs-pDNA [containing 10 μg pDNA (GFP)] in serum-free and antibiotic-free medium for 5 h. Then, medium was remover, and the cells were cultured in DMEM with 10% fetal bovine serum for 48 h. Meanwhile, cells were transfected with pDNA (GFP) using Lipofectamine 2000 as positive control; and cells without treatment were served as normal control. Lastly, cells were observed under inverted fluorescence microscope. This experiment has got the approval of the animal experimental ethics committee of Cangzhou Central Hospital.

### Intracellular distribution assay

Rat chondrocytes were treated with SLNs-pDNA for 4 h, and stained with Lyso-Tracker Red (staining for lysosome) for 30 min. Lastly, cells were observed under laser scanning confocal microscope.

### qRT-PCR

Total RNA from cells was obtained by Trizol (Invitrogen) following the manufacturer's instructions. PrimeScript™ RT reagent Kit (Takara, Dalian, China) was utilized to obtain cDNA by reverse transcription of RNA. The qRT-PCR was carried out by the SYBR Premix Ex Taq TM II (Takara). The PCR primers are shown as following: integrin β1 sense primer: 5’- ACTTCTCCTGTGTCCGCTACAAG-3’ and antisense primer: 5’-GGTGTCAGTACGCGTGGTACA-3’; and glyceraldehyde-3-phosphate dehydrogenase (GAPDH) sense primer: 5'-GTGGATCAGCAAGCAGGAGT-3' and antisense primer: 5'-AAAGCCATGCCAATCTCATC-3'. GAPDH was served as the internal control. Lastly, mRNA expression data was evaluated by 2-ΔΔCt method.

The article "Cationic solid lipid nanoparticles loaded by integrin β1 plasmid DNA attenuates IL-1β-induced apoptosis of chondrocyte" was retracted in 2023. Reasons: plagiarized images; duplicated images; overlap with other authors' work; signs of a paper mill.

### Cell viability assay

CCK-8 method was used to evaluate cell viability. To evaluate the cytotoxicity of SLNs-pDNA, rat chondrocytes were grown in 96-well plates and treated with 10 μL of SLNs-pDNA with different doses (1, 4, 8, 20, and 30 μg), respectively. Meanwhile, cells were transfected with pDNA (GFP) using Lipofectamine2000 as positive control; and cells without treatment were served as normal control. Moreover, to investigate the effect of SLNs-pDNA on cell viability in inflammatory injury model, rat chondrocytes with or without inflammatory injury were treated with SLNs-pDNA. After conventional incubation for 24 h, each well was added with 10 μl of CCK-8 (Dojindo Molecular Technologies, Inc., Kumamoto, Japan) for another 1.5 h. Lastly, microplate spectrophotometer was used to evaluate cell viability based on the absorbances at 450 nm.

### 5-bromo-2′-deoxy-uridine (BrdU) assay

BrdU kit (Invitrogen) was used for cell proliferation detection. Specifically, rat chondrocytes were treated according to the above design for 48 h, followed by incubation of BrdU by another 40 min. Following treatment with 4% paraformaldehyde to fix cells for 15 min away from light, cell immunofluorescence was carried out using anti-BrdU antibody, and DAPI was used for the staining of nucleus. The cells were observed under inverted microscope (Olympus, Japan), and the images were used to calculate the percentage of BrdU-positive cells.

### Mitochondrial membrane potential detection

Mitochondrial membrane potential depolarization was detected using commercial JC-1 kit (Beyotime). At high membrane potential, JC-1 shows red fluorescent aggregates; while JC-1 presents green fluorescent monomers at low membrane potential. Briefly, rat chondrocytes were treated according to the above design for 24 h, and then stained with 1 ml of JC-1 dye at 37°C for 20 min. Next, cells were rinsed with JC-1 buffer, and observed under an inverted microscope (Olympus, Japan).

### Cell apoptosis assay

FITC-Annexin V Apoptosis kit was used in this experiment. Rat chondrocytes were treated according to the above design. Trypsin was used to digest rat chondrocytes, and then the cells were harvested. Next, cells were rinsed with PBS, and resuspended with Binding Buffer. After the incubation of FITC-Annexin V and PI with cells for 15 min, flow cytometer (BD, CA, USA) was used to calculate the number of apoptotic cells.

The article "Cationic solid lipid nanoparticles loaded by integrin β1 plasmid DNA attenuates IL-1β-induced apoptosis of chondrocyte" was retracted in 2023. Reasons: plagiarized images; duplicated images; overlap with other authors' work; signs of a paper mill.

### Western blotting assay

Rat chondrocytes were treated according to the above design. The collected cells were lysed by RIPA lysis buffer (Gibco), and then proteins were extracted by commercial kit (Pierce, Rockford, IL, USA). Next, after resolved on PAGE gel, protein sample was transferred to PVDF. Afterwards, the membrane was blocked, and reacted with integrin β1, pro-caspase-3, pro-caspase-9, cleaved caspase-3, cleaved caspase-9 or β-actin primary antibody (1:300, Santa Cruz) overnight at 4°C. After the incubation with second antibody (1:5000, Jackson, USA), the protein levels were detected by enhanced chemiluminescence (ECL, Millipore, USA).

### Statistical analysis

Data were presented as the mean ± SD. One-way ANOVA followed by multiple comparison was used for data comparisons based on SPSS software. P < 0.05 was considered significant.
